This article has been retracted.

# Mechanisms of M2 Macrophage-Derived Exosomal Long Non-coding RNA PVT1 in Regulating Th17 Cell Response in Experimental Autoimmune Encephalomyelitisa

**DOI:** 10.3389/fimmu.2020.01934

**Published:** 2020-09-04

**Authors:** Lei Wu, Jinjin Xia, Donghui Li, Ying Kang, Wei Fang, Peng Huang

**Affiliations:** ^1^Department of Neurology, The Second Affiliated Hospital of Zhejiang, University School of Medicine, Hangzhou, China; ^2^Department of Neurology, Changxing Hospital, Second Affiliated Hospital of Medical College of Zhejiang University, Huzhou, China; ^3^Department of Pollution Source Statistics, Zhejiang Provincial Environmental Monitoring Center, Hangzhou, China; ^4^School of Pharmacy, Anhui University of Traditional Chinese Medicine, Hefei, China

**Keywords:** experimental autoimmune encephalomyelitis, M2 macrophages, exosomes, long non-coding RNA PVT1, microRNA-21-5p, SOCS5

## Abstract

Long non-coding RNA (lncRNA) is pivotal for multiple sclerosis (MS), but the potential mechanism of lncRNA PVT1 in MS animal model, experimental autoimmune encephalomyelitis (EAE) still remains unclear. In this study, macrophages were firstly isolated and induced to polarize into M2 macrophages. M2 macrophage-derived exosomes (M2-exos) were extracted and identified, and EAE mouse model was established and treated with M2-exos. The effect of M2-exos on EAE mice was evaluated by clinical scores. The proportion of Treg and Th17 cells in spinal cord cells and splenocytes, and levels of inflammatory factors were measured. The targeting relationships among PVT1, miR-21-5p, and SOCS5 were verified. The expression of JAKs/STAT3 pathway-related proteins was measured. After M2-exo treatment, the clinical score of EAE mice decreased, and demyelination and inflammatory infiltration improved; Th17 cells decreased, Treg cells increased, and the levels of inflammatory factors decreased significantly. SOCS5 and PVT1 were downregulated and miR-21-5p was upregulated in EAE mice. PVT1 could sponge miR-21-5p to regulate SOCS5. SOCS5 alleviated EAE symptoms by repressing the JAKs/STAT3 pathway. Together, M2-exos-carried lncRNA PVT1 sponged miR-21-5p to upregulate SOCS5 and inactivate the JAKs/STAT3 pathway, thus reducing inflammation and protecting EAE mice. This study may offer novel treatments for MS.

## Introduction

Experimental autoimmune encephalomyelitis (EAE) is an acknowledged animal model for multiple sclerosis (MS), and it is evidenced that CD4^+^ T cells, releasing interleukin (IL)-17, namely T helper (Th)17 cells, link with EAE pathogenesis (1). EAE is an intricate disease where the interactions of various immune and neurological pathological mechanisms contribute to demyelination, inflammation, axonal loss, and gliosis, the key features of MS, leading to central nervous system (CNS) tissue damage (2). EAE animals are characterized with demyelination, fatigue, handicapped axonal conduction, blurred vision, progressive paralysis, cognitive deficits, and weight loss (3, 4). McFarl and HF et al. evidenced the involvement of Th17, CD8^+^ and regulatory T (Treg) cells in MS induction, and noted that peripheral T cells produced inflammatory cytokines and probably differentiated on activation into Th1 and Th17 cells (5). Besides, in demyelinating lesions, the interaction between macrophages and CD4^+^ T cells is implicated in MS pathobiology (6). M2 macrophages are alternatively activated macrophages, and predominantly inhibit immune responses (7). Emerging evidence has revealed the beneficial roles of M2 macrophages in ameliorating EAE, and macrophages M2 polarization blocks EAE progression, which is associated with subsequent inhibition of proinflammatory Th1 and Th17 cells both in peripheral lymph system and CNS (8). In light of this, we try to explore the underlying mechanism of M2 macrophages in Th17 cells balance in EAE.

Exosomes containing proteins, RNA, lipids, and metabolites, can be engulfed by local tissues or released into body fluid to affect distant target organs, and exosomes are critical in intercellular communication in physiological and pathological conditions (9). It is believed that M2 macrophage-derived exosomes (M2-exos) transfer certain proteins or signals to tumor cells to regulate their migration (10). Specific long non-coding RNAs (lncRNAs) are preferentially packaged into exosomes, and the abundance of exosomal lncRNA correlates with their expression in the original cells (11). The lncRNA plasmacytoma variant translocation 1 (PVT1), located at 8q24.21, is recognized as an oncogene in diverse cancers, whose aberrant expression is proven to relate to cancer development (12). Interestingly, Eftekharian et al. identified a significant downregulation of PVT1 in relapsing-remitting MS (RRMS) patients (13). It is recognized that PVT1 functions as a competing endogenous (ce)-RNA in the miR-mediated interaction-network toward the microRNA (miR)-200 family (14). It is suggest that increased methylation in miR-21 associates with lower expression of mature miR-21 in CD4^+^ T cells of RRMS patients (15). Suppressor of cytokine signaling (SOCS) family proteins are rapidly transcribed in response to intracellular JAK-STAT signaling, a cascade regulator of cytokine-induced immune response (16). SOCS3 and SOCS5 are mainly expressed in Th2 and Th1 cells, respectively, and they reciprocally inhibit Th1 and Th2 differentiation processes (17). SOCS5 is downregulated in the serum of MS patients (18). From all above, it is reasonable to hypothesize that there are interactions between M2-exos-carried lncRNA PVT1, miR-21-5p, and SOCS5 in EAE. Thus, a string of experiments were performed in this study to justify the hypothesis.

## Materials and Methods

### Ethics Approval and Informed Consent

This study along with the animal experiments was approved and supervised by the ethics committee of Zhejiang University School of Medicine. Great efforts were made to minimize the animals and their affliction.

### Isolation and Culture of Mouse Macrophages

Specific pathogen-free grade mice (purchased from Beijing Vital River Laboratory Animal Technology Co., Ltd, Beijing, China, SYXK (Hu) 2017-0014) were euthanized by cervical dislocation. The mice were intraperitoneally injected with 5 mL pre-cooled serum-free Roswell Park Memorial Institute (RPMI)-1640 medium, with the abdomen gently rubbed for 2–3 min. After 5 min, the peritoneum was lifted with tweezers, the peritoneal lavage fluid was sucked by a straw, and the peritoneal lavage was repeated once. The supernatant was discarded via centrifugation at 4°C, and the precipitated cells were suspended in RPMI1-640 medium (containing 100 U/mL penicillin, 100 μg/mL streptomycin and 10% fetal bovine serum, FBS). After counting, the cell concentration was adjusted to 2 × 10^6^ cells/mL/well in 24-well plates, and cells were cultured at 37°C with 5% CO_2_. After 2–4 h, the medium was renewed, other non-adherent cells were discarded, and the adherent monolayer cells were macrophages.

### Induction and Identification of M2 Macrophages

As mentioned above, macrophages were incubated in the complete medium, and M2 expression was obtained by incubation for 24 h with 20 ng/mL mouse IL-4 (Sigma-Aldrich, Merck KGaA, Darmstadt, Germany) (19). Macrophages were collected, suspended with 5 μL phosphate buffered saline (PBS), dripped on the slide, and added with Wright's dye solution after drying. Next, macrophages were mixed with buffer solution at 1:2, dyed for 10 min, washed under running water, and observed under the microscope after natural drying. For flow cytometry, samples (1 × 10^6^) to be tested were collected and suspended, and added with 2 μL fluorescent antibodies and homologous control. Then samples were incubated on ice for 30 min, washed with fluorescence-activated cell sorting buffer, and fixed with 10% formalin. Finally, the positive rate of antigen was determined using a flow cytometer. The antibodies were CD68 (1:100, ab31630, Abcam, Cambridge, MA, USA) and CD163 (1:60, ab182422, Abcam).

### Preparation of Conditioned Medium (CM) and Isolation and Identification of M2 Macrophage-Derived Exosomes (M2-exo)

Polarized macrophages were cultivated in RPMI1-640 medium supplemented with 100 U/mL penicillin, 100 μg/mL streptomycin, and 10% FBS without exosomes (centrifuged at 200,000 g for 18 h for exosome depletion). The supernatant was collected at 700 g centrifugation for 10 min and served as CM (M2-CM).

The exosomes were separated from M2-CM by differential ultracentrifugation. After PBS washing, exosomes were pre-fixed with 2.5% glutaraldehyde in PBS (pH 7.4) for 2 h and fixed again with 1% osmium tetroxide in PBS for another 2 h. The exosomes were incubated on a glow-discharged copper grid for 1 min, and stained with a drop of 2% phosphotungstic acid aqueous solution. Afterwards, the excess buffer was carefully drained from the edge of the copper grid with filter papers. The mesh was dyed with 2% uranyl acetate (pH 7.0) for 40 s. The samples were air-dried at room temperature and examined under the transmission electron microscope (TEM) at 80 keV. The exosomes were diluted into 1 mL in tris(pyrazolyl)methane for further analysis. ZetaView PMX 110 (Particle Metrix GmbH, Microtrac, Meerbusch, Germany) was applied to measure the size and concentration of exosomes using Nanosight Tracking Analysis. The levels of exosome-specific markers CD63 (1: 1000, ab59479), CD81 (1: 1000, ab79559) and tumor susceptibility gene 101 (TSG101, 1: 1000, ab30871) (all purchased from Abcam) were detected with western blot analysis.

### Cell Transfection

The si-lncRNA PVT1 and si-lncRNA negative control (NC) vectors were synthesized by Shanghai Integrated Biotech Solutions Co., Ltd (Shanghai, China). According to the instructions of the kit, si-lncRNA PVT1 and si-lncRNA NC were mixed with Dharmafect Duo (Dharmacon, Thermo Scientific, Waltham, MA, USA), and then co-cultured with M2 macrophages, followed by extraction of the exosomes.

### EAE Model Establishment and Grouping

C57BL/6 mice (12 weeks, 20–25 g) (Beijing Vital River Laboratory Animal Technology Co., Ltd., Beijing, China) were fed in separate ventilated cages with adequate food and water.

After anesthesia and intraperitoneal injection of an anesthetic mixture consisting of tiletamine and xylazine (10 mL/kg), EAE was induced with myelin pligodendrocyte glycoprotein (MOG)35-55 peptide (MEVGWYRSPFSRVVHLYRNGK; % peak area by HPLC ≥ 95, AnaSpec, EGT Corporate Headquarters, Fremont, CA, USA). Mice were subcutaneously injected with the emulsion (300 μL/flank) concluding 300 μg MOG35-55 in PBS and an equal amount of complete Freund's adjuvant composed of 300 μg heat-killed *mycobacterium tubercolosis* H37Ra (Difco Laboratories, Sparks, MD, USA). After that, the mice were intraperitoneally injected with 100 μL pertussis toxin (500 ng/100 μL) (Sigma-Aldrich), and the injection was repeated 48 h later. EAE was accompanied by a progressive process of degeneration with obvious pathological signs, including tail limpness and loss of movement in the hind leg. At the 28th day after EAE-induction, all mice were euthanized by intraperitoneal injection of Tanax (5 mL/kg body weight). Spinal cords and spleen tissues were processed to assess disease parameters.

Mice were randomized into normal group (*n* = 24, without any treatment), EAE group (*n* = 18, at the time of disease onset, about 14 days after immunization, EAE mice were injected with PBS via tail vein, 5 μL/mouse), EAE + M2-CM group (*n* = 18, at the time of disease onset, EAE mice were injected with M2-CM via tail vein, 5 μL/mouse), EAE + M2-exo group (*n* = 24, at the time of disease onset, EAE mice were injected with M2-exo via tail vein, 150 μg/mouse), M2-si-lncRNA NC-exo group (*n* = 18, at the time of disease onset, EAE mice were injected with M2-si-lncRNA NC-exo via tail vein, 150 μg/mouse), M2-si-lncRNA PVT1-exo group (*n* = 18, at the time of disease onset, EAE mice were injected with M2-si-lncRNA PVT1-exo via tail vein, 150 μg/mouse), miR-21-5p mimic group (*n* = 18, at the time of disease onset, EAE mice were injected with miR-21-5p mimic via tail vein, 50 μg/mouse), and miR-21-5p inhibitor group (*n* = 18, at the time of disease onset, EAE mice were injected with miR-21-5p inhibitor via tail vein, 50 μg/mouse). In each group, six mice were randomly selected for pathological section, six for reverse transcription quantitative polymerase chain reaction (RT-qPCR) and western blot analysis, six for splenocyte and spinal cord cell isolation and subsequent experiments, and the other for biodistribution experiments.

### Clinical Disease Score

Each mouse was graded blind every 2 days and recorded a clinical score ranging from 0 to 4. The standard for mouse scoring was as follow. No significant changes in motor function vs. non-immunized mice (score 0), flabby tip of tail (score 0.5), flabby tail (score 1.0), flabby tail and hind leg inhibition (score 1.5), flabby tail and hind legs weakness (score 2.0), flabby tail and hind legs dragging (score 2.5), flabby tail and complete paralysis of hind legs (score 3.0), flabby tail, complete paralysis of hind legs and partial paralysis of front legs (score 3.5), and minimal movement and alert (score 4.0).

### Histopathological Examination

After the mice were euthanized, the lumbar enlargement of spinal cords was embedded in paraffin, sliced into serial sections at 5 μm, and one section was taken at intervals of 100 μm. Six sections of each tissue were taken for hematoxylin and eosin (HE) staining.

The luxol fast blue (LFB) staining was applied for determination of myelin differentiation. Spinal cord sections from mice that received PBS or exosomes were dehydrated for 1 h and then washed with ethanol, lithium carbonate, Harris hematoxylin, acid alcohol, ammonium hydroxide, and eosin separately. Six mice (at least 10 sections per mouse) were utilized for LFB staining. Multiple sections from at least 6 different spinal cord regions of 6 mice were used to quantify myelinated and unmyelinated axons. All spinal cord sections were assessed under the microscope (Nikon, Tokyo, Japan).

### RT-qPCR

The one-step method of TRIzol (Invitrogen, Carlsbad, CA, USA) was employed to extract total RNA, and extracted high-quality RNA was confirmed using ultraviolet analysis and formaldehyde denaturation electrophoresis. RT-qPCR was conducted as per the instructions of a RT-qPCR kit (Thermo Fisher Scientific, Shanghai, China) with glyceraldehyde-3-phosphate dehydrogenase as an internal reference for CCL22, peroxisome proliferator-activated receptor gamma (PPARγ), PVT1, and SOCS5, while U6 as an internal reference for miR-21-5p. PCR primers were provided by Shanghai Sangon Biotechnology Co., Ltd. (Shanghai, China) (Table 1). The amplification and dissolution curves were confirmed after the reaction, and data were analyzed by 2^−ΔΔ*Ct*^ method.

**Table 1:** Primer sequences of RT-qPCR.

**Gene**	**Primer sequence**
miR-21-5p	F: 5′-TAGCTTATCAGACTGATGTTGA-3′
	R: 5′-TCAACATCAGTCTGATAAGCTA-3′
GAPDH	F: 5′-GGGAGCCAAAAGGGTCAT-3′
	R: 5′-GAGTCCTTCCACGATACCAA-3′
U6	F: 5′-CGCTTCGGCAGCACATATAC-3′
	R: 5′-AATATGGAACGCTTCACGA-3′
CCL22	F: 5′-ATTACGTCCGTTACCGTCTG-3′
	R: 5′-TAGGCTCTTCATTGGCTCAG-3′
PPARγ	F: 5′-GCCTTGCAGTGGGGATGT-3′
	R: 5′-CTCGCCTTTGCTTTGGTC-3′
PVT1	F: 5′-GATGCCCCTCAAGATGGCTG-3′
	R: 5′-GACACGAGGCCGGCCACGC-3′
SOCS5	F: 5′-ATAAAGTGGGAAAAATGTGG-3′
	R: 5′-TTGCCTTGACTGGTTCTCGT-3′

*RT-qPCR, reverse transcription quantitative polymerase chain reaction; miR, microRNA; GAPDH, glyceraldehyde-3-phosphate dehydrogenase; PPARγ, peroxisome proliferator-activated receptor gamma; PVT1, plasmacytoma variant translocation 1; SOCS5, suppressor of cytokine signaling 5; F, forward; R, reverse*.

### Biodistribution Experiments

M2-exo labeled with lipophilic DiR dye was perfused into the tail vein. In detail, 4 μL DiR dye was added to 1 mL Diluent C (fluorescent cell linker kit for general cell membrane labeling; Sigma-Aldrich, No. CGLDIL-6 × 10 mL) 5 min before incubation with exosomes or the control. Next, 2 mL bovine serum albumin (1%, BSA) was added, and exosome samples were filtered with 300 kDa Vivaspin filters (Sartorius Stedim Biotech GmbH, Goettingen, Germany) by centrifugation at 4,000 g. Then samples were washed with 5 mL PBS in triplicate. The same volume of dye was used as the control in all experiments. EAE and wild-type (WT) mice were observed and photographed at the 3 and 24 h using an intelligent visual inspection system (IVIS, Perkin-Elmer, Waltham, MA, USA) with a highly sensitive charged coupled device camera to image the high wavelength fluorescence. Mice were euthanized at the 24 h, and organs were imaged at both time points. Mice were sedated with isoflurane and real-time imaged via 1–2 min exposure with indocyanine green (ICG) filter at 745 nm excitation. After each real-time imaging, the mouse organs were isolated and imaged via 1–2 second exposure (ICG filter at 745 nm excitation). Fluorescence for each mouse and organ image was quantified using live imaging software in IVIS.

### Splenocyte Preparation

After the mice were euthanized, the spleens were taken out and cut off with ophthalmic scissors. Then spleen tissues were ground repeatedly with a 2-mL glass injection needle on 200-mesh cell sieves and washed with RPMI-1640 solution. Then the splenocyte suspension was collected into a sterile cell culture dish. If Th17 cells were detected subsequently, the splenocytes were gently mixed and then added into 24-well plates, with 500 μL splenocyte suspension in each well. At the same time, the sterile MOG35-55 solution (10 μg/mL) was added for re-immunization stimulation at 37°C with 5% CO_2_. Afterwards, splenocytes were added with flow cytological stimulants Phorbol 12-myristate 13-acetate (50 ng/mL), Ionomycin (500 ng/mL) and Brefeldin A (3 ug/mL) after 8 h. Cell culture medium was collected after incubation for 14 h in a CO_2_ constant-temperature incubator. The splenocytes were centrifuged at 1,900 g for 10 min to discard the supernatant and the splenocytes were suspended in normal saline and collected into a one-time flow cytometry tube for flow cytometry detection (about 10^6^ cells per tube). If Th17 was not detected, the cells were centrifuged and collected directly into the flow tube.

### Spinal Cord Cell Isolation (20)

After the mice were euthanized, the spine was cut at the top of the column, and the spinal cord was compressed with a sterile 1 × DPBS hydraulic pressure by a No. 21 needle. Tissues were homogenized and passed through a 70-μm nylon cell strainer (Millipore, Z742103-50EA) with 10 15 mL sterile 1 × DPBS containing 0.2% glucose (Millipore, G7528) into 50-mL conical tubes. The homogenate was centrifuged at 600 × g for 6 min. The supernatant was decanted and the pellet was resuspended in 6-mL sterile 70% SIP. Afterwards, the resuspended homogenate was moved to a sterile 15-mL polypropylene conical tube and 3 mL sterile 50% SIP was layered over. Another 3 mL sterile 35% SIP was layered on the top of the 50% SIP layer, and 2 mL sterile 1 × DPBS was layered on the top of the 35% layer. Next, the prepared 15 mL conical tubes were centrifuged at 2,000 × g for 20 min without brake. Three discrete layers were established after centrifugation. The top layer of myelin was removed and cells from the interface between 70–50% SIP and 50–35% SIP were collected in separate conical tubes. After that, isolated cells were resuspended in sterile 1 × DPBS and centrifuged at 600 × g for 6 min to remove any remaining percoll. Then cells were immediately subjected to downstream applications. If Th17 cells were detected, the treatment was consistent with the above treatment of splenocytes. In the 24-well plate and sterile MOG35-55 solution, re-immune stimulation was carried out. After 8 h, flow cytometry stimulant was added to culture the cells for 14 h, and then flow cytometry was carried out. If Th17 cells were not detected, cells were centrifuged directly and collected into flow tube.

### Flow Cytometry

For Th17 cell detection, the above collected splenocytes or spinal cord cells were prepared into single cell suspension according to flow cytometry, about 10^6^ cells per tube. CD4 antibody (0.25 μL) labeled with fluorescence was put into each tube and incubated for 30 min without exposure to light. The fluorescent labeled IL-17A antibody (1:250, ab79056, Abcam) was added to the fixed membrane breaker and buffer after proper treatment, and incubated at room temperature for 60 min without exposure to light. Next, cells were resuspended with fixed membrane breaker buffer, and centrifuged to discard the supernatant. Finally, cells were resuspended with 2 mL flow staining solution and loaded on the flow cytometer.

For Treg cell and T cell detection, the collected splenocytes or spinal cord cells were prepared into single cell suspension according to flow cytometry, about 10^6^ cells per tube. Treg cells were detected via CD4 (1:250, ab59474, Abcam), CD25 (1:250, ab210330, Abcam) and Foxp3 (1:250, ab210232, Abcam) antibodies, and T cells were detected by CD4 and CD8 (1:250, ab22378, Abcam) antibodies according to Th17 detection procedures.

### Dual Luciferase Reporter Gene Assay

PVT1 fragment containing the binding site of miR-21-5p was cloned into the pmirGLO oligosaccharide enzyme vector (Promega, Madison, WI, USA), and the pmirGLO-PVT1-WT reporting vector was constructed. The pmirGLO-PVT1-mutant type was constructed with the mutant binding site of miR-21-5p based on pmirGLO-PVT1-Wt. After that, the constructed vectors were transfected into macrophages and then co-transfected with miR-21-5p mimic and miR-NC, respectively. After 48 h, the luciferase activity was assessed using dual luciferase reporter gene assay system (Promega, Madison, WI, USA), and the relative activity was calculated as the ratio of firefly luciferase activity to renilla luciferase activity.

### Western Blot Analysis

The proteins were extracted to determine the concentration as per the instructions of a bicinchoninic acid kit (Thermo Scientific Pierce, Rockford, IL, USA). The extracted proteins were boiled and run on sodium dodecyl sulfate polyacrylamide gel electrophoresis from 80 to 120 v. Afterwards, the proteins were transferred into the polyvinylidene fluoride membranes (Millipore Corp., Billerica, MA, USA). The membranes were blocked and incubated with primary antibodies at 4°C overnight: SOCS5 (1:1000, ab97283, Abcam), Janus kinase 1 (JAK1, 1:1000, ab47435, Abcam), p-JAK1 (1:1000, ab138005, Abcam), signal transducer and activator of transcription 3 (STAT3, 1:5000, ab119352, Abcam) and p-STAT3 (1:2000, ab76315, Abcam). Then the membrane was rinsed in tris-buffered saline tween (TBST), and cultured for 1 h with secondary antibody (ZSGB-BIO, Beijing, China) labeled by horseradish peroxidase. After TBST washing, the proteins were visualized by enhanced chemiluminescence reagent and developed by Gel EZ imager (Bio-Rad Laboratories, CA, USA). Finally, the target bands were analyzed with Image J software (National Institutes of Health, Bethesda, Maryland, USA) for gray value analysis.

### Enzyme-Linked Immunosorbent Assay (ELISA)

Levels of mouse tumor necrosis factor-α (TNF-α, MTA00B, R&D Systems, Minneapolis, MN, USA), IL-17 (M1700, R&D Systems), IL-6 (M6000B, R&D Systems), and IL-1β (MLB00C, R&D Systems) were detected as per the instructions of different Quantikine ELISA kits.

### Statistical Analysis

The data were analyzed with SPSS 21.0 statistical software (IBM Corp., Armonk, NY, USA) and checked in normal distribution with the Kolmogorov-Smirnov test. The measurement data are exhibited as mean ± standard deviation. Comparisons between two groups were analyzed using *t*-test, among multiple groups were evaluated using one-way or two-way analysis of variance (ANOVA), and pairwise comparisons after ANOVA were conducted by Tukey's multiple comparisons test. The *p*-value was calculated by a two-tailed test and *p* < 0.05 inferred a statistical difference.

## Results

### Identification of M2 Macrophages

Macrophages were obtained from the abdominal cavity of mice. After primary culture, the cells were stained by Wright's staining. Under the microscope, the macrophages were in irregular shape, the nucleus was dark blue, mostly biased to one side, and showed typical morphological characteristics of macrophages (Figure 1A). The macrophage specific molecular markers CD68 and CD163 were positive detected by flow cytometry (Figure 1B). M2 macrophages were prepared by IL-4 induction. M2 macrophages were obviously enlarged under the microscope, mainly exhibiting as larger round cells (Figure 1C). RT-qPCR was used to detect the typical polarization molecules CCL22 and PPARγ in non-classically activated macrophages (M2). It was found that mRNA expression of CCL22 and PPARγ increased significantly after induction (both *p* < 0.05; Figures 1D–E), indicating that M2 macrophages were successfully induced and obtained.

**Figure 1:** M2 macrophages are successfully induced and obtained. **(A)** Representative image of macrophage morphology detected by Wright's staining; **(B)** The macrophage specific molecular markers CD68 and CD163 were positive detected by flow cytometry; **(C)** Representative images of the morphology of macrophage and M2 macrophage under an optical microscope; **(D,E)** RT-qPCR was used to detect the typical polarization molecules CCL22 and PPARγ. vs. the blank group, ***p < 0.001. Data were analyzed with the *t*-test. Repetitions = 3.

### M2 Macrophage Derived-Exosomes Protect EAE Mice

EAE mice were induced by MOG35-55. About 14 days later, the mice reached the peak of disease and their tails and hind limbs were completely paralyzed and their postures were flat. Each mouse was graded every other day and the clinical score was assigned to 0–4. Among them, score 0 was for healthy WT mice and score 4 was for dead mice, as we mentioned in the method. To study the role of M2 macrophages in EAE, we injected M2-CM into EAE mice. Compared with the control mice injected with PBS, M2-CM could significantly improve the clinical score (Figure 2A).

**Figure 2:** M2-exos protect EAE mice. **(A)** Clinical score of EAE mice treated with PBS, M2-CM, or M2-exo; **(B)** Observation of the morphology and size of M2-exos by TEM; **(C)** Exosome concentration and particle size by Nanosight Tracking Analysis; **(D)** Detection of exosome markers CD63, CD81, and TSG101 by western blot analysis; **(E)** Detection of demyelination in spinal cord sections using LFB staining; **(F)** Pathological examination of spinal cord sections in mice detected by HE staining; **(G)** T cell infiltration into the spinal cord of EAE mice detected with flow cytometry. Compared with the PBS group, **p < 0.01, ***p < 0.001. Data are analyzed with two-way ANOVA, and Tukey's multiple comparisons test was utilized for *post hoc* test *n* = 6.

The exosomes were separated from M2-CM. The exosome morphology was observed under the TEM (Figure 2B). The average size of exosomes was about 100 nm (Figure 2C). The expression of exosome markers CD63, CD81, and TSG101 was positive in these vesicles (Figure 2D). Injection of M2-exo into EAE mice showed that M2-exo improved the clinical score of EAE mice as M2-CM did (Figure 2A).

Demyelination is one of the markers of MS and eventually leads to clinical symptoms (21). Similarly, the clinical symptoms of EAE mice are also related to spinal cord demyelination (2). Therefore, to analyze the severity of demyelination in EAE mice, we used LFB to analyze the myelin sheath in spinal cord sections of EAE mice treated with different methods. Compared with the PBS-treated mice, the degree of demyelination in spinal cord sections of M2-exo-treated mice was decreased (Figure 2E).

Early MS lesions are characterized by focal infiltration of monocytes and lymphocytes into the brain and spinal cord (22). Through the HE staining, we observed that the inflammatory infiltration of spinal cord sections in EAE mice was significantly improved after treatment with M2-exo (Figure 2F). T cell infiltration into CNS is another marker of neuroinflammation, especially in MS (23). Therefore, we also used flow cytometry to assess T cell infiltration into spinal cord of EAE mice. The percentage of CD4^+^ and CD8^+^ infiltration in spinal cord of M2-exo-treated mice was significantly reduced relative to that of PBS-treated mice (*p* < 0.05; Figure 2G). Briefly, M2-exos protected EAE mice.

### LncRNA PVT1 Enters EAE Mice From M2-exos

MS is a chronic immune-regulated CNS disease. Recently, abnormal expression of lncRNA is reported as a potential cause of MS, and it found that PVT1 was markedly downregulated in MS patients (13). By using lipophilic dye DiR labeling, it displayed that exosomes mainly existed in the liver and spleen of mice after tail vein injection, and fluorescence also existed in the spinal cord after M2-exo entered the EAE mice, demonstrating M2-exos were associated with EAE (Figure 3A). PVT1 expression in spinal cord of EAE mice was detected by RT-qPCR. Compared with healthy mice, PVT1 expression in spinal cord of EAE mice was evidently downregulated (*p* < 0.05), while in M2-exo-treated mice was higher than that in EAE mice (*p* < 0.05; Figure 3B). To further confirm that lncRNA PVT1 entered EAE mice through M2-exo, we transfected si-lncRNA PVT1 into M2 macrophages and then isolated the exosomes. PVT1 expression in M2-si-lncRNA PVT1-exo was reduced (Figure 3C). After M2-si-lncRNA PVT1-exo was injected into EAE mice, PVT1 expression in EAE mice reached the lowest level (Figure 3B). These results suggested that lncRNA PVT1 entered EAE mice from M2-exos.

**Figure 3:** LncRNA PVT1 enters EAE mice from M2-exos. **(A)** DiR labeled exosomes were traced in mice. It showed that exosomes mainly existed in liver and spleen 24 h after they entered the mice. Fluorescence also appeared in spinal cord of EAE mice; **(B,C)** Relative PVT1 expression in spinal cord of EAE mice with different treatment detected by RT-qPCR. Compared with the blank group, ***p < 0.001; compared with the EAE group, *##p* < 0.01, *###p* < 0.001. Data in **(B)** are analyzed with one-way ANOVA, and Tukey's multiple comparisons test was utilized for *post hoc* test. Data in **(C)** were analyzed by the *t*-test *n* = 6.

### LncRNA PVT1 Carried by M2-exo Inhibits Th17 Cell Proinflammatory Response in EAE Mice

Treg deficiency promotes spontaneous autoimmune disease in mice, and restoring Treg function can hinder EAE (24). Flow cytometry showed that Treg cells (CD4^+^ CD25^+^ FOXP3^+^) in spinal cord cells of EAE mice was expressly lower than that of normal mice (*p* < 0.05), and markedly increased under the action of M2-exo (*p* < 0.05), while it was the lowest under the action of M2-si-lncRNA PVT1-exo (*p* < 0.05). The number of Treg cells (CD4^+^ CD25^+^ FOXP3^+^) in splenocytes was the same as that in spinal cord cells (Figure 4A).

**Figure 4:** LncRNA PVT1 inhibits the proinflammatory response induced by Th17 cells in EAE mice. **(A,B)** Detection of Treg and Th17 cells in spinal cord cells and splenocytes by flow cytometry; **(C)** Detection of inflammatory factors in spinal cord cells by ELISA. Compared with the blank group, ***p < 0.001; compared with the EAE group, #*p* < 0.05, *##p* < 0.01, *###p* < 0.001. Data are analyzed with two-way ANOVA, and Tukey's multiple comparisons test was utilized for *post hoc* test *n* = 6.

Several inflammatory T cell subsets, like Th1 and Th17, especially Th17, are key drivers of EAE (25, 26). Therefore, we detected Th17 in EAE mice by flow cytometry. It showed that Th17 (CD4^+^ IL-17A^+^) in spinal cord cells of EAE mice increased (*p* < 0.05), decreased significantly after M2-exo treatment (*p* < 0.05), and reached the highest level after M2-si-lncRNA PVT1-exo treatment (*p* < 0.05). The trend in splenocytes was consistent with that in spinal cord cells (Figure 4B).

Afterwards, we measured the inflammatory factors TNF-α, IL-17, IL-6, and IL-1β in spinal cord. Compared with normal mice, the levels of inflammatory factors increased in EAE mice, decreased significantly under the action of M2-exo, but the levels of inflammatory factors in EAE mice were elevated after M2-si-lncRNA PVT1-exo treatment (all *p* < 0.05; Figure 4C). These results indicated that lncRNA PVT1 inhibited the proinflammatory response induced by Th17 cells in EAE mice.

### LncRNA PVT1 Competitively Binds to miR-21-5p and Upregulates SOCS5 Expression in EAE Mice

Through literature review, we found that silencing miR-21-5p can effectively interfere with the Th17 cell differentiation to treat EAE (27). In our previous experiments, M2-exo was found to reduce the clinical score of EAE mice, and the carrying PVT1 inhibited the proinflammatory response induced by Th17. We suspected that there may be a targeting relationship between lncRNA PVT1 and miR-21-5p. Through the database (http://starbase.sysu.edu.cn, https://cm.jefferson.edu/rna22/Interactive/) search verification and dual-luciferase reporter gene assay, we found that there is indeed a targeting relationship between lncRNA PVT1 and miR-21-5p (Figures 5A,B). Besides, RT-qPCR demonstrated that miR-21-5p expression increased in spinal cord of EAE mice, decreased in spinal cord of M2-exo-treated mice and further increased in M2-si-lncRNA PVT1-exo-treated mice (all *p* < 0.05; Figure 5D).

**Figure 5:** LncRNA PVT1 competitively binds to miR-21-5p and upregulates SOCS5 expression in EAE mice. **(A)** Database (http://starbase.sysu.edu.cn, https://cm.jefferson.edu/rna22/Interactive/) analysis of binding relationship between lncRNA PVT1 and miR-21-5p, together with miR-21-5p, and SOCS5; **(B,C)** Targeting relationship between lncRNA PVT1 and miR-21-5p, together with miR-21-5p, and SOCS5 detected by dual-luciferase reporter gene assay, compared with the NC group, ***p < 0.001; **(D)** Relative miR-21-5p expression in spinal cord of EAE mice with different treatment detected by RT-qPCR; **(E,F)** mRNA and protein levels of SOCS5 in spinal cord of EAE mice with different treatment detected by RT-qPCR and western blot analysis. Compared with the blank group, ***p < 0.001; compared with the EAE group, #*p* < 0.05, *###p* < 0.001. Data in **(D–F)** are analyzed with one-way ANOVA, in **(B,C)** are and analyzed with two-way ANOVA, Tukey's multiple comparisons test was utilized for *post hoc* test *n* = 6.

SOCS family proteins are important in MS progression, among which SOCS1 and SOCS5 are significantly downregulated in the serum of MS patients (18). According to the analysis of database (http://starbase.sysu.edu.cn), there were binding sites between miR-21-5p and SOCS5 (Figure 5A). Similarly, we validated the targeting relationship between miR-21-5p and SOCS5 via dual-luciferase reporter gene assay (Figure 5C). It showed that miR-21-5p could target SOCS5. Then we detected SOCS5 levels in EAE mice, and found SOCS5 levels were significantly downregulated in spinal cord of EAE mice (*p* < 0.05), but upregulated in spinal cord of EAE mice treated with miR-21-5p inhibitor (Figures 5E,F).

### miR-21-5p Targets SOCS5 to Inhibits Th17 Cell Proinflammatory Response in EAE Mice via the JAKs/STAT3 Pathway

After verifying the targeting relationship between lncRNA PVT1 and miR-21-5p, and miR-21-5p and SOCS5, we wanted to further study the mechanism of SOCS5 in EAE. We injected miR-21-5p mimic and miR-21-5p inhibitor into EAE mice by the tail vein alone or with exosomes to observe the disease situation of EAE mice. It exhibited that clinical scores were enhanced in EAE mice with single injection of miR-21-5p mimic, while reduced in EAE mice with miR-21-5p inhibitor injection (all *p* < 0.05; Figure 6A).

**Figure 6:** SOCS5 alleviates EAE symptoms by inhibiting pro-inflammatory response of Th17 cells through the JAKs/STAT3 pathway. **(A)** Clinical scores of EAE mice with different treatment; **(B)** Levels of JAKs/STAT3 pathway-related proteins and their phosphorylation levels in EAE mice detected by western blot analysis; vs. the blank group, ***p < 0.001; compared with the EAE group, #*p* < 0.05, *##p* < 0.01, *###p* < 0.001; **(C,D)** Detection of Treg and Th17 cells in spinal cord cells and splenocytes by flow cytometry; compared with the EAE group, *p < 0.05, **p < 0.01, ***p < 0.001; **(E)** Detection of inflammatory factors in spinal cord cells by ELISA; compared with the EAE group, *p < 0.05, **p < 0.01, ***p < 0.001. Data are analyzed with two-way ANOVA, and Tukey's multiple comparisons test was utilized for *post hoc* test *n* = 6.

According to western blot analysis, the phosphorylation levels of JAK1 and STAT3 were significantly increased in EAE mice, and further enhanced in EAE mice injected with miR-21-5p mimic alone, while reduced in EAE mice with miR-21-5p inhibitor injection (all *p* < 0.05; Figure 6B). Flow cytometry detected Th17 and Treg cells in spinal cord cells and splenocytes, and found that Th17 cells in EAE mice with low SOCS5 expression (EAE group and miR-21-5p mimic group) were greatly higher than those in EAE mice with high SOCS5 expression (EAE + M2-exo group and miR-21-5p inhibitor group), while Treg cells were the opposite (Figures 6C,D). ELISA showed that SOCS5 expression was negatively correlated with levels of inflammatory factors in spinal cord cells. The levels of inflammatory factors in mice with high SOCS5 expression (miR-21-5p inhibitor group) were substantially lower than that in mice with low SOCS5 expression (EAE group, miR-21-5p mimic group) (Figure 6E). It concluded that SOCS5 alleviated EAE symptoms by inhibiting pro-inflammatory response of Th17 cells through the JAKs/STAT3 pathway.

## Discussion

In the late stage of EAE, M2 macrophages are correlated with anti-inflammatory response and tissue repair, and become dominant in the CNS, leading to the recovery of homeostasis and improvement of physical functions and increase of immunoregulatory expression of lesions in EAE model (28, 29). Inspired by these reporters, we hypothesized there existed a ceRNA interaction involving M2-exos-carrying lncRNA PVT1 and miR-21-5p in EAE. Collectively, we came to a conclusion that lncRNA PVT1/miR-21-5p/SOCS5 axis was protective for EAE through the JAKs/STAT3 pathway.

First, we claimed that M2-exo improved the clinical score of EAE mice, and decreased demyelination and percentage of CD4^+^ and CD8^+^ infiltration in the spinal cord. MS is characterized by inflammatory infiltrating CD4^+^ and CD8^+^ T cells, and CD8^+^ T cells constitute major lymphocytes in MS lesions (30). Anti-CD4 abolished EAE when given prior to the first immunization, and antibody-mediated CD8^+^ T cell exhaustion before EAE induction aggravated clinical disease (31). What's more, transgenic mice with deficient functional CD8^+^ T cells displayed severe myelin pathology, axonal injury, inflammation, and exacerbated tissue destruction after EAE induction (32). Transferring of M2 macrophages could reduce the severity of clinical signs of EAE by inhibiting T cell proliferation (33). Thereby, M2-exo protected against EAE.

Additionally, this study demonstrated that lncRNA PVT1 expression in EAE mice was significantly downregulated, and increased after M2-exo treatment. Consistent observation of lncRNA PVT1 downregulation in RRMS patients may indicate the potential therapeutic effects of PVT1 in MS (13). Our study also found that lncRNA PVT1 carried by M2-exo inhibited the proinflammatory response induced by Th17 cells in EAE mice, by increasing Treg cells (CD4^+^ CD25^+^ FOXP3^+^) and decreasing Th17 (CD4^+^ IL-17A^+^) and inflammatory factors TNF-α, IL-17, IL-6, and IL-1β in spinal cord cells and splenocytes. Treg lymphocyte secretes anti-inflammatory cytokines and is implicated in EAE remission (34). CD4^+^ CD25^+^ Foxp3^+^ naturally occurring Treg cells are effective inhibitors of major immune responses and protector of immunological homeostasis and self-tolerance (35). Indeed, downregulation of Th1 and Th17 responses was beneficial in MS (2). Th17 cells secrete proinflammatory cytokines, including IL-17A, IL-22, and IL-21, and IL-17 production directly contributes to EAE severity (36). Induced Treg contributed to T self-tolerance in EAE by repressing the proliferation and function of antigen-specific encephalitogenic T cells (37).

Furthermore, miR-21-5p expression was increased, while SOCS5 was downregulated in EAE mice. miR-21 was upregulated in peripheral blood mononuclear cells of RRMS patients in relapse (38, 39). miR-21 was upregulated in Th17-stimulated T cells, and silencing miR-21 may be an effective treatment for MS and other Th17-mediated autoimmune diseases (41). Meanwhile, another study revealed that SOCS1 and SOCS5 expression was noticeably reduced in RRMS patients (18). SOCS5 accumulation led to inhibition of STAT1 and STAT3 and the promotion of differentiation of CD4^+^ cells into Th1 and Th17 (proinflammatory cytokine secreting cells) (40). Meanwhile, this present study indicated that M2-exosomal lncRNA PVT1 competitively bound to miR-21-5p and upregulated SOCS5 expression in EAE mice. Corroborating evidence supported that macrophages-derived exosomes could also release miR-21 inhibitor to gastric cancer cells and inhibit their migration (42). Moreover, we found that SOCS5 alleviated EAE symptoms by inhibiting proinflammatory response of Th17 cells through the JAKs/STAT3 pathway. STAT3 in CD41 and CD81 T cells was activated in the early stage of inflammatory diseases, reflecting proinflammatory response (43). STAT3 is an essential Th17 differentiation-specific protein, and is necessary for differentiation of CD4^+^ T cells to Th17 cell in EAE (44). Evidence has claimed that blockade of the JAK/STAT pathway was anticipated to offer therapeutic immunosuppression and anti-inflammation, and thus provide treatments for autoimmune diseases (45). Strikingly, M2 macrophages lightened the severity of atypical EAE, which was related to inhibited STAT3 activation and macrophage activation, diminished Th17 expression, and reduced leukocyte infiltration (46).

## Conclusions

Taken together, these results offer insights into the mechanism of M2-exosomal lncRNA PVT1 and its ceRNA network in EAE development, whereby M2-exo-carrying lncRNA PVT1 alleviated inflammation induced by Th17 cells in EAE mice, and lncRNA PVT1 competitively bound to miR-21-5p, upregulated SOCS5 expression and inhibited the JAKs/STAT3 pathway. The exosome-mediated intercellular communication between M2 macrophages and PVT1 or miR-21-5p-treated spinal cord cells enriches our understanding of EAE. However, MS affects various human activities with wide psychological, social and economic impacts, none of which could be modeled properly in EAE mouse models (2). Thus, further study should be conducted to find out the possible applicable approach for MS in the clinical setting based on results obtained from this study. However, for the cells that may be lost when washing the plate, we think they cannot guarantee the stable transformation of M2 during M2 induction, and will cause certain interference to our research, so these cells are not in the research of our manuscript. We will carry out further research on this part of cells in the future.

## Data Availability Statement

All datasets presented in this study are included in the article.

## Ethics Statement

This study along with the animal experiments was approved and supervised by the ethics committee of Zhejiang University School of Medicine.

## Author Contributions

All authors listed, have made substantial, direct and intellectual contribution to the work, and approved it for publication.

## Conflict of Interest

The authors declare that the research was conducted in the absence of any commercial or financial relationships that could be construed as a potential conflict of interest.
